The article "Clinical Effect of Fuzheng Guben Decoction in the Treatment of Localized Prostate Cancer and Its Influence on Immune Function under Continuous Nursing Intervention" was retracted in 2023. Reasons: signs of a paper mill; suspected computer-generated content; unreliable results or conclusions; concerns about the data.

# Clinical Effect of Fuzheng Guben Decoction in the Treatment of Localized Prostate Cancer and Its Influence on Immune Function under Continuous Nursing Intervention

**DOI:** 10.1155/2022/3472722

**Published:** 2022-09-16

**Authors:** Yanling Zhou, Lan Liu, Lifei Gao

**Affiliations:** ^1^Yiwu Fuyuan Hospital, Yiwu 322200, China; ^2^Department of Obstetrics, Department Nursing, West China Second University Hospital, Sichuan University/West China School of Nursing, Sichuan University, Chengdu 610041, China; ^3^PLA General Hospital Jingxi Medical District of the Same Level of Outpatient Department, Comprehensive Internal Medicine, Beijing 100144, China

## Abstract

In order to explore the clinical effect and immune function of patients with localized prostate cancer combined with continuous nursing intervention and Fuzheng Guben decoction, a total of 72 patients with prostate cancer admitted to our hospital from January 2020 to June 2021 are selected and analyzed. The patients are randomly divided into a study group and control group randomly, and the control group and the research group are treated with routine intervention and chemotherapy, continuous nursing intervention, and Fuzheng Guben decoction on the basis of chemotherapy, respectively. The incidence of postoperative urinary incontinence and other complications between the two groups are counted, and the differences of FHIT, CatD, CatL, CD68, and CD83 levels in the patients are compared. Furthermore, the total treatment response rate and self-attitude score of the two groups are compared after treatment. The experimental results demonstrate that the total effective rate and self-attitude score of patients in the study group are significantly better than those in the control group.

## 1. Introduction

Among all male malignant tumors, prostate cancer has a high incidence rate in the world. In recent years, the incidence rate of prostate cancer in China has increased significantly [1]. This disease often occurs in elderly men aged 60–80 years, and the incidence rate increases with age [2]. Urinary incontinence is the most common postoperative complication after prostatectomy, usually lasting about 1 year after surgery [3]. Therefore, continuous nursing intervention is very important for these patients. The nursing intervention plan can continue to provide coordinated and effective medical and nursing services for patients in hospital and after discharge, and play an important role in stabilizing the condition and improving the prognosis of patients [4]. Chemotherapy is a common clinical treatment method after prostatectomy for prostate cancer, which has a significant therapeutic effect. However, this method will cause great damage to the patient's body, and it is easy to cause the patient's immune function to decline and damage the liver and kidney function. This has a great negative impact on the prognosis of patients [5]. Studies have shown that traditional Chinese medicine (TCM) is used to improve the prognosis of tumor patients. Patients taking Fuzheng Jiejian decoction can improve the damaged body function and have great advantages in detoxification and diuresis [6]. Especially for the damage caused by chemotherapy, it can effectively improve the treatment effect of cancer and bring some improvement to patients [7].

The article "Clinical Effect of Fuzheng Guben Decoction in the Treatment of Localized Prostate Cancer and Its Influence on Immune Function under Continuous Nursing Intervention" was retracted in 2023. Reasons: signs of a paper mill; suspected computer-generated content; unreliable results or conclusions; concerns about the data.

According to the clinical research data, continuous nursing intervention combined with Fuzheng Guben decoction in the treatment of localized prostate cancer is rarely reported. The purpose of this paper is to discuss the continuity nursing intervention bottom allied with the centralizer thrift soup treatment of the localized prostate cancer clinical effect and the influence on immune function in patients. It is clearly evident that continuity nursing intervention under the application of the centralizer thrift soup for localized prostate cancer can obtain a better clinical effect and improve the patient's immune function significantly.

This paper is organized as follows: Section 2 presents the related work and Section 3 illustrates the data and proposed methods. In Section 4, the results and analysis are presented. Some concluding remarks are made in Section 5.

## 2. Related Work

At present, surgical treatment has a good effect on the spread of prostate cancer. However, some scholars believe that surgical treatment will also have different degrees of adverse effects on patients. It mainly includes the following: hormone balance, sexual dysfunction, urinary incontinence, and other complications, as well as fatigue and gastrointestinal discomfort [8, 9]. In addition, patients also have physical pain and greater psychological stress [10]. Zraik and Heß-Busch [11] indicated that radiotherapy and chemotherapy can cause serious damage to the patient's body and result in nausea, abdominal pain, headache, alopecia, and anemia, though help prolong the survival period. Therefore, it is particularly important to carry out continuous intervention and nursing for patients. Patients can receive continuous and targeted nursing measures during hospitalization and after discharge. The professional intervention work of medical personnel can be extended from the hospital to the patients' families, which is the systematic extension and transfer service of nursing work [12]. Traditional Chinese medicine also plays an important role in the injury caused by radiotherapy and chemotherapy.

The article "Clinical Effect of Fuzheng Guben Decoction in the Treatment of Localized Prostate Cancer and Its Influence on Immune Function under Continuous Nursing Intervention" was retracted in 2023. Reasons: signs of a paper mill; suspected computer-generated content; unreliable results or conclusions; concerns about the data.

By establishing personal files for patients, continuous nursing intervention can provide targeted nursing for different patients, and carry out continuous nursing intervention for patients through various intervention methods, such as nursing plan arranged for patients before discharge, continuous follow-up and rehabilitation exercise guidance for patients after discharge, and psychological counseling within the family [13]. Various forms of continuous intervention broke through the traditional intervention methods and realized the continuity of nursing work on the boundary of time and space. For hospitalized patients, the details of diet, medication, and reasonable exercise in daily life can be recorded in detail. In addition, patients need regular follow-up and appointment after discharge. During the monthly follow-up, the patients were asked about their recent physical recovery, review status, and whether there were related complications, and the relevant information of the patients was timely mastered and recorded. In addition, patients were urged to spend more time with their families and friends, and actively socialize to eliminate the psychological burden and pressure of patients and ensure a positive psychological state. By establishing a patient group, it can help patients to adopt correct rehabilitation methods and pay attention to rational medication. In addition, it can also promote the interaction between patients and medical personnel, patients and patients, and strengthen the communication between patients and medical workers. Through reasonable guidance and arrangement, the patients received pelvic floor muscle function training after discharge to help the patients recover [14]. Through the explanation of prostate cancer cases, medical staff can make patients better grasp the rehabilitation knowledge and reduce the incidence of adverse complications after training. Patients can share their experiences with their families and other patients, share their psychological status, and help patients build confidence to overcome the disease [15]. Fuzheng Guben decoction can obtain good clinical efficacy, which includes the decoction from grass, Fritillaria, Jujube, Paeonia alba, Pinellia ternata, Astragalus membranaceus, American ginseng, tangerine peel, and *Angelica sinensis*. In modern pharmacological studies, Xianxin Astragalus can strengthen the adrenal cortex function of patients and has an obvious effect on killing tumor cells and promoting their apoptosis. The overall prescription has a significant effect on improving the patient's body, alleviating the damage of chemotherapy, improving the patient's immunity, and prolonging the patient's survival time.

The article "Clinical Effect of Fuzheng Guben Decoction in the Treatment of Localized Prostate Cancer and Its Influence on Immune Function under Continuous Nursing Intervention" was retracted in 2023. Reasons: signs of a paper mill; suspected computer-generated content; unreliable results or conclusions; concerns about the data.

FHIT genes can induce apoptosis, while CatL and CatD are a class of invasive genes, mainly existing in lysosomes, which have a strong hydrolysis effect on proteins in the extracellular matrix and can destroy the structure of the extracellular matrix, thus accelerating tumor cells to break through the extracellular matrix and infiltrate surrounding tissues [16, 17]. Thus, it is necessary to study whether Fuzheng Guben decoction combined with chemotherapy can increase the expression of tumor suppressor genes or weaken the occurrence of invasive genes. In the view of traditional Chinese medicine, Fuzheng Jianjian decoction has the functions of nourishing Yin, transforming Qi, and supplementing blood. Modern pharmacological studies have shown that Fuzheng Jianjian decoction, including amino acids, naphtha, saponins, steroids, polysaccharides, organic acids, has a more significant effect on inhibiting tumor cell proliferation and gene expression, and can also effectively inhibit the growth of tumor cells [18]. CD83 can play a role on the surface of DC and is a kind of a landmark molecule which can inhibit the stimulating activity of T cells through DC, weaken the proliferation of T cells, and play an important role in the immune response of DC.CD68 is a transmembrane glycoprotein expressed on mononuclear macrophages, and the antigen treated by this cell can activate T cells, thereby promoting a series of immune responses, and playing a role in inhibiting tumor growth and promoting immune function enhancement [19]. Fuzheng Guben decoction plays an important role in promoting the expression of CD68 and CD83, and improving the immune function of patients. Also, it can effectively reduce the level of invasive genes in prostate cancer patients, enhance the expression level of tumor suppressor genes and CD68, CD83, and enhance the immune system function of patients [20].

## 3. Data and Proposed Methods

### 3.1. General Information

A total of 72 prostate cancer patients admitted to our hospital from January 2020 to June 2021 are selected as the research subjects and are randomly divided into a study group and control group by the random number table method, with 36 patients in each group. Patients in the study group ranged in age from 64 to 69 years, with an average age of 66.54 ± 2.83 years. The mean course of the disease is 3.27 ± 0.91 years. Marital status: 1 case is single, 35 cases are married; there are 6 cases in stage 1, 10 cases in stage 2, 13 cases in stage 3 and 7 cases in stage 4. Prostate cancer volume <60 mL in 19 cases, ≥60 mL in 17 cases. Low differentiation, medium differentiation, and high differentiation are 6, 17, and 13 cases, respectively. There are 16 cases with lymph node metastasis and 20 cases without lymph node metastasis. The age range of control group is 62–70 years, with an average age of 65.84 ± 3.91 years. The mean course of disease is 2.97 ± 1.13 years. Marital status: unmarried 2 cases and married 34 cases. There are 7 cases in stage 1, 9 cases in stage 2, 14 cases in stage 3, and 6 cases in stage 4. 20 patients with prostate cancer volume <60 mL and 16 patients with prostate cancer volume ≥60 mL. Among them, low differentiation, medium differentiation and high differentiation are 8, 15, and 13 cases, respectively. There are 13 cases with lymph node metastasis and 23 cases without lymph node metastasis. There is no significant difference in baseline data between the two groups (*p* > 0.05), indicating comparability. This study is approved by the ethics committee of our hospital, and all patients gave informed consent and signed informed consent. Inclusion criteria are as follows: (1) patients diagnosed with prostate cancer by pathological examination of our hospital; (2) the patient does not suffer from serious underlying diseases; (3) the education level of the patients is above primary school; (4) patients are in a good mental state and can cooperate with the study. Exclusion criteria are as follows: (1) illness aggravation or other systemic complications during the study period; (2) taking other drugs to treat patients during the intervention period; (3) the patient also suffers from other malignant tumors; (4) poor patient compliance.

The article "Clinical Effect of Fuzheng Guben Decoction in the Treatment of Localized Prostate Cancer and Its Influence on Immune Function under Continuous Nursing Intervention" was retracted in 2023. Reasons: signs of a paper mill; suspected computer-generated content; unreliable results or conclusions; concerns about the data.

### 3.2. Methods

The control group is given conventional chemotherapy drugs, cisplatin for injection (Qilu Pharmaceutical Co., Ltd., National drug approval H37021357, batch No. 1204015, specification: 20 mL/20 mg) 100 mg/m2+ fluorouracil for injection (Hainan Zhuotai Pharmaceutical Co., Ltd., National drug approval H20051627, batch No. 20130826, specification: 0.5 g/dose) 1 g/m^2^ 7 days intravenously as a course of treatment. Patients continued to take medicine after 1 week of withdrawal in the middle of every 2 courses. Both groups of patients are continuously treated for 1 month. In terms of nursing intervention, health education manuals are issued to patients after discharge to guide their diet and medication arrangements and matters needing attention, emphasizing the content of rehabilitation training. Patient are instructed to have a review at the specified time, and the intervention time is 3 months after discharge.

Patients in the study group carried out continuous intervention in nursing. Specific measures are as follows: (1) personal files are set up when patients are discharged from hospital and personal information such as mailing address and contact information is reserved. Whether follow-up endocrine-related treatment is carried out after surgery and whether adverse reactions occurred during hospitalization are recorded to form a complete continuous intervention file; (2) a continuing intervention group is established, which is led by the head nurse and attending physician. The group members are trained and required to master the related treatment and postoperative care of adenocarcinoma; (3) before the patients are discharged, the team members gave detailed guidance on the matters needing attention of the patients' care and informed the appointment method of the return visit clinic to make patients understand the content and significance of rehabilitation follow-up; (4) the first follow-up is conducted on the second day after the first discharge, with the frequency of follow-up being 1 to 2 times per month. During the follow-up, the patient's personal condition after discharge and return visit are understood; (5) in the follow-up, the focus must be on understanding the patient's physical recovery and whether complications and other content are present. The patient must be instructed to carry out rehabilitation training and be sure to comply with the doctor's advice. At the same time, communicate with patients to understand whether adverse reactions occurred during the medication period, and register in the patient's personal files; (6) use a WeChat group to send patients and their families the relevant knowledge about adenocarcinoma care, in terms of dietary considerations and scientific exercise. In the group, send text, pictures, videos, and other ways to help patients understand postoperative rehabilitation knowledge and reasonable rehabilitation training. Patiently answer patients' questions and help them form a good health consciousness. Organize patient exchange so that patients exchange experience in the recovery process, to build confidence to overcome the disease. It can be guided by the attending physician to conduct pelvic floor muscle training to improve the professional degree.

The article "Clinical Effect of Fuzheng Guben Decoction in the Treatment of Localized Prostate Cancer and Its Influence on Immune Function under Continuous Nursing Intervention" was retracted in 2023. Reasons: signs of a paper mill; suspected computer-generated content; unreliable results or conclusions; concerns about the data.

In addition, patients in the study group and the control group received the same chemotherapy regimen, and are treated with Fuzheng Guben decoction in parallel. The prescriptions include the following: decoction of *Codonopsis pilosula* 20 g, Caulis spatholobus 20 g, licorice 6 g, tangerine peel 9 g, *Pinellia ternata* I2 g, dried ginger 9 g, *Herba membranaceus* I5 g, Fructus ligustris lucidum 15 g, Xue Jiao 9 g, Atractylodes adactylies macrocephala 30 g, and Poria cocos 12 g with 400 ml water and extract 300 ml. Take 1 dose a day separately twice in the morning and evening, take with warm water. The duration of 2 weeks is 1 cycle, and 4 consecutive cycles are taken.

### 3.3. Observation Indicators and Inspection Standards

#### 3.3.1. Comparison of Urinary Incontinence between the Study Group and Control Group

The International Urinary Incontinence Advisory Committee Urinary Incontinence Questionnaire (ICI-Q-LF) is conducted to investigate the urinary incontinence of the patients and scored them according to three aspects, namely, the degree of impact of urinary incontinence on life, frequency of urinary incontinence, and quantity of urine leakage. 1 score is basically no influence on patients' life, 3 score is certain influence, and 5 score is serious influence. The frequency of urinary incontinence in patients is 1 point once per week, 3 points 2–3 times per week, and 5 points more than once per day. In terms of urine leakage, 1 score is given for incontinence with a small amount of urine exudating, 3 score for a large amount of urine exudating, and 5 score for complete urine outflow.

#### 3.3.2. Comparison of the Incidence of Complications

The number of complications such as infection, abdominal distention, nausea, and vomiting during the recovery period is recorded. The total incidence can be calculated by the following formula: total incidence = (number of infection + number of abdominal distention + number of nausea and vomiting)/total number of patients.

#### 3.3.3. Comparison of the Overall Immune Function of Patients

The expression levels of tumor suppressor genes and invasive genes in the two groups after treatment are compared. The mRNA expression levels of the fragile histidine triad gene (FHIT) and the mRNA expression levels of invasion-related genes cathepsin D (CatD) and cathepsin L (CatL) are detected by polymerase chain reaction (PCR). The LineGene 9600 plus produced by Hangzhou Bori Technology Co., Ltd. is used for testing in strict accordance with the operating instructions.

To compare the expressions of CD68 and CD83 in peripheral blood of patients in the two groups before and after treatment, blood is collected in a fasting state in the morning before and after treatment in patients in the two groups, and the levels of CD68 and CD83 in patients are detected by FACScalibur flow cytometry using a FC500 flow cytometer of Beckman strictly follow the instructions for testing.

#### 3.3.4. Comparison of Treatment Effect

The total effective rate of the treatment is counted. Clinical recovery is manifested as pain in sexual organs and/or disappearance of cancer pain or great relief when urinating or erecting, and the number of conventional cancer cells in prostate massage fluid is less than 15/HP. The significant effect is pain in sexual organs and/or relief of cancer pain in patients when urinating and erecting. The number of conventional cancer cells in prostate massage fluid is 15 to 20/HP. Effective performance is sexual organ pain and/or is in urination, erection, patients with cancer pain significantly relieved, and the number of conventional cancer cells in prostate massage fluid is 20 to 30/HP; ineffective performance is pain in sexual function organs and/or is in urination, erection patients cancer pain feeling no significant improvement, and the number of conventional cancer cells in prostate massage fluid is unchanged.

The article "Clinical Effect of Fuzheng Guben Decoction in the Treatment of Localized Prostate Cancer and Its Influence on Immune Function under Continuous Nursing Intervention" was retracted in 2023. Reasons: signs of a paper mill; suspected computer-generated content; unreliable results or conclusions; concerns about the data.

#### 3.3.5. Comparison of Self-Attitude Assessment

The self-efficacy information of patients can be collected and evaluated by the Self-Efficacy Scale. The Self-Efficacy Scale includes the dimensions of mitigation self-evaluation, positive attitude, and self-determination content, and is divided with a total of 28 related items. The evaluation score of each item is arranged from 1 to 5 points, which corresponds to “no confidence,” “there is a little bit of faith,” “confident,” “more confident,” and “very confident.” The total score is equal to 140, which is positively correlated with good self-efficacy.

### 3.4. Statistical Methods

SPSS 26.0 statistical software is used to analyze the data of this study. The measurement data of normal distribution is expressed as ($\bar{x}$ ± *s*), and the *t*-test is used to compare the two samples. The count data are represented by the number of cases and percentage, using the *x*^*2*^ test and using *p* < 0.05 is a statistical difference.

## 4. Results and Analysis

### 4.1. Comparison of Urinary Incontinence between the Study Group and Control Group

The improvement of urinary incontinence in the study group is better than that in the control group, and the difference is statistically significant (*p* < 0.05), as shown in Table 1 and Figure 1.

### 4.2. Comparison of the Occurrence of Complications between the Study and Control Groups

The total incidence of complications in the study group is lower than that of the control group, with significant differences (*p* < 0.05), as shown in Table 2.

### 4.3. Content of Tumor Suppressor Genes and Invasion Genes in the Study and Control Groups

The expression of tumor suppressor gene FHIT is more obvious in the study group than that in the control group, and the expression of invasion gene CatL and CatD are weaker than that in the control patients, *p* < 0.05, as shown in Table 3 and Figure 2.

### 4.4. CD68 and CD83 Expression in the Peripheral Blood of the Study and Control Groups

Before treatment, CD68 and CD83 expressions are insignificant, *p* > 0.05. After treatment, their expression increased in both groups, with *p* < 0.05, while the levels of CD68 and CD83 in the study group are significantly higher than those in the control group, with *p* < 0.05, as shown in Table 4 and Figures 3, and 4.

The article "Clinical Effect of Fuzheng Guben Decoction in the Treatment of Localized Prostate Cancer and Its Influence on Immune Function under Continuous Nursing Intervention" was retracted in 2023. Reasons: signs of a paper mill; suspected computer-generated content; unreliable results or conclusions; concerns about the data.

### 4.5. Comparison of Patient Efficacy between the Two Patient Groups

Efficacy of the study group and control group is significantly better than that of the control group, with significant statistical differences, *p* < 0.05, as shown in Table 5.

### 4.6. Comparison of Self-Attitude Assessment between the Study Group and Control Group

On admission, there is no significant difference in the scores of self-efficacy in all dimensions between the two groups (*p* < 0.05); three months after discharge, the scores of self-efficacy in all dimensions in both groups increased, and the scores of self-efficacy in all dimensions in the observation group are higher than those in the control group, with a statistical significance (*p* < 0.05), as shown in Table 6, Figures 5 and 6.

## 5. Conclusions

In this study, the clinical effect and immune function of patients with localized prostate cancer combined with continuous nursing intervention and Fuzheng Guben decoction is explored. The experimental results reveal the application of Fuzheng Guben decoction under continuous nursing intervention can significantly promote the postoperative recovery of prostate cancer patients. Their urinary incontinence symptoms are significantly improved, and the related complications are also significantly reduced. It is also found that the contents of tumor suppressor gene FHIT and immune cells CD68 and CD83 are significantly increased, and the expression of invasive genes CatD and CatL is significantly decreased. Besides, the immune function of the patients is significantly recovered. The self-attitude score of the patients is better, the psychological burden of the patients is significantly reduced, which is also of great value to the prognosis of the patients and worthy of clinical application. It should be noted that the clinical effect of the combined intervention scheme has not been demonstrated by other researchers, and the number of objects is relatively small in this study. Therefore, the follow-up should expand the sample size to further explore the clinical value of the joint scheme, so as to provide a more effective treatment for patients with prostate cancer.

## Figures and Tables

**Figure 1:** Urinary incontinence condition.

**Figure 2:** Expression of total tumor suppressor genes and invasion genes.

**Figure 3:** CD68 and CD83 expression in peripheral blood before treatment.

The article "Clinical Effect of Fuzheng Guben Decoction in the Treatment of Localized Prostate Cancer and Its Influence on Immune Function under Continuous Nursing Intervention" was retracted in 2023. Reasons: signs of a paper mill; suspected computer-generated content; unreliable results or conclusions; concerns about the data.

**Figure 4:** CD68 and CD83 expression in peripheral blood after treatment.

**Figure 5:** Comparison of the self-efficacy scores at hospital admission.

**Figure 6:** Comparison of self-efficacy scores at 3 months from discharge.

**Table 1:** Comparison of urinary incontinence between the two groups [$\bar{x}$ *±* *s*, points].

Group	Example number (*n*)	The degree of impact on life	The degree of impact on life	Missing urine volume	Total points
The research group	36	2.57 ± 0.88	1.83 ± 0.92	2.01 ± 0.56	6.35 ± 1.53
Control group	36	3.72 ± 1.23	2.91 ± 1.21	2.51 ± 0.77	9.31 ± 2.11
*t*		−4.562	−4.263	−3.151	4.195
*p*		<0.001	<0.001	0.002	0.010

**Table 2:** Comparison of the occurrence of complications in the two groups [*n* (%)].

Group	Example number (*n*)	Infect	Abdominal distension	*N* and *V*	Total incidence
The research group	36	1 (2.77)	1 (2.77)	2 (5.55)	4 (11.11)
Control group	36	3 (8.33)	2 (5.55)	4 (11.11)	9 (25.00)
*x* ^*2*^					4.251
*p*					0.030

**Table 3:** Expression of total tumor suppressor genes and invasion genes in the two groups ($\bar{x}$ *±* *s*).

Group	Example number (*n*)	FHIT	CatL	CatD
The research group	36	1.61 ± 0.24	0.61 ± 0.17	0.71 ± 0.11
Control group	36	1.11 ± 0.22	0.91 ± 0.24	0.94 ± 0.20
*t*		14.573	9.495	10.913
*p*		0.001	0.001	0.001

**Table 4:** Comparison of peripheral blood CD68 and CD83 expression in the two groups (%, $\bar{x}$ *±* *s*).

Group study group (*n* = 36)	CD68		CD83	
	Pretherapy	Post-treatment	Pretherapy	Post-treatment
Control group (*n* = 36)	2.91 ± 0.87	10.23 ± 3.01^*∗*^	1.74 ± 0.53	5.09 ± 1.54^*∗*^
Group	2.86 ± 0.91	3.13 ± 1.21^*∗*^	1.82 ± 0.56	2.32 ± 0.91^*∗*^
*t*	0.613	22.813	0.924	16.987
*p*	0.531	0.001	0.317	0.001

*Note.* Compared with this group before treatment, ^*∗*^*p* < 0.05.

**Table 5:** Comparison of patient efficacy between the two patient groups [*n* (%)].

Group	Example number(*n*)	Clinical recovery	Excellence	Effective	Invalid	Total effective rate
The research group	36	8 (22.22)	10 (27.78)	12 (33.33)	6 (16.67)	30 (83.33)
Control group	36	6 (16.67)	7 (19.44)	11 (30.56)	12 (33.33)	24 (66.67)
*x* ^*2*^						3.951
*p*						0.020

**Table 6:** Comparison of self-efficacy scores between the two groups ($\bar{x}$ ± *s*).

Group	Self-decision making		Positive attitude		Self-decompression		Total efficiency score	
	On admission	3 months after discharge	On admission	3 months after discharge	On admission	3 months after discharge	On admission	3 months after discharge
Control group (*n* = 36)	7.32 ± 2.02	13.31 ± 0.77^*∗*^	31.21 ± 2.49	39.57 ± 3.12	20.11 ± 0.67	31.77 ± 2.01	67.32 ± 6.01	84.62 ± 5.13
Study group (*n* = 36)	7.19 ± 1.12	17.68 ± 0.59^*∗*^	30.78 ± 1.88	45.76 ± 2.13	20.11 ± 0.59	36.97 ± 1.99	68.44 ± 5.51	89.99 ± 3.80
*t*	0.338	-27.029	-0.827	9.831	0.000	11.031	-0.824	5.047
*p*	0.737	<0.001	0.411	<0.001	1.000	<0.001	0.413	<0.001

*Note.* Compared with the current group on admission, ^*∗*^*p* < 0.05.

The article "Clinical Effect of Fuzheng Guben Decoction in the Treatment of Localized Prostate Cancer and Its Influence on Immune Function under Continuous Nursing Intervention" was retracted in 2023. Reasons: signs of a paper mill; suspected computer-generated content; unreliable results or conclusions; concerns about the data.

## Data Availability

The simulation experiment data used to support the findings of this study are available from the corresponding author upon request.

## References

[1] Taneja S. (2018). Re: surveillance or metastasis-directed therapy for oligometastatic prostate cancer recurrence: a prospective, randomized, multicenter phase II trial. *The Journal of Urology*.

[2] Alwhaibi A., Alsanea S., Almadi B., Al-sabhan J., Alosaimi F. D. (2022). Androgen deprivation therapy and depression in the prostate cancer patients: review of risk and pharmacological management. *The Aging Male*.

[3] Hoeh B., Wenzel M., Müller M. (2022). Urethral sphincter length but not prostatic apex shape in preoperative MRI is associated with mid-term continence rates after radical prostatectomy. *Diagnostics*.

[4] Wild K., Sharma N., Mattek N., Karlawish J., Riley T., Kaye J. (2021). Application of in-home monitoring data to transition decisions in continuing care retirement communities: usability study. *Journal of Medical Internet Research*.

[5] Mota J. M., Barnett E., Nauseef J. (2019). Platinum-based chemotherapy in metastatic prostate cancer with alterations in DNA damage repair genes. *Journal of Clinical Oncology*.

[6] He J., Xie H. L., Zhang P. H. (2022). Clinical study of fuzheng guben decoction combined with acupoint injection in the treatment of chemotherapy related nausea and vomiting of malignant tumor. *New traditional Chinese medicine*.

[7] Ciprut S., Sedlander E., Watts K. L. (2018). Designing a theory based intervention to improve the guideline-concordant use of imaging to stage incident prostate cancer. *Urologic Oncology: Seminars and Original Investigations*.

[8] Adam S., Feller A., Rohrmann S., Arndt V. (2018). Correction to: health-related quality of life among long-term (≥5 years) prostate cancer survivors by primary intervention: a systematic review. *Health and Quality of Life Outcomes*.

[9] Scherr K., Delaney R. K., Ubel P. (2022). Preparing patients with early stage prostate cancer to participate in clinical appointments using a shared decision making training video. *Medical Decision Making*.

[10] Diefenbach M. A., Benedict C., Miller S. M. (2018). Examining the impact of a multimedia intervention on treatment decision-making among newly diagnosed prostate cancer patients: results from a nationwide RCT. *Translational Behavioral Medicine*.

[11] Zraik I. M., Heß-Busch Y. (2021). Management of chemotherapy side effects and their long-term sequelae. *Urologe Ausgabe A*.

The article "Clinical Effect of Fuzheng Guben Decoction in the Treatment of Localized Prostate Cancer and Its Influence on Immune Function under Continuous Nursing Intervention" was retracted in 2023. Reasons: signs of a paper mill; suspected computer-generated content; unreliable results or conclusions; concerns about the data.

[12] Turns B., Springer P. R., Sibley D. S. (2019). Removing the ‘mystery’ in therapy: transparency as a continuous intervention in family psychotherapy. *Journal of Family Psychotherapy*.

[13] Huffman C., van Gameren E. (2018). The roll-out of a health insurance program and its impact on the supply of healthcare services: a new method to evaluate time-varying continuous interventions. *International Journal for Equity in Health*.

[14] Lu X. Y., Liang Z., Hu M. Y. (2022). Curative effect of pelvic floor muscle exercise on urinary incontinence after radical prostatectomy-Comparisons of different approaches at different time point. *Andrologia*.

[15] Su H. C., Shen Y. J., Lin G. W. (2019). Attitudes of prostate cancer patients towards postoperative penile rehabilitation and their influencing factors. *National Journal of Andrology*.

[16] Park S., Bennett-Baker P., Ahmed S. (2021). Locus-specific transcription silencing at the FHIT gene suppresses replication stress-induced copy number variant formation and associated replication delay. *Nucleic Acids Research*.

[17] Yin S. E., Hu J. G., Jiang Z. C. (2021). Cathepsin D deficiency in RPE cells mediates stargardt disease pathogenesis. *Investigative Ophthalmology & Visual Science*.

[18] Wei P. F., Yang Y. Y., Huang H. (2018). Efficacy and safety of Fuzheng gubentang combined with intensity modulated radiotherapy in the treatment of cervical cancer. *Jilin Traditional Chinese Medicine*.

[19] Silva J. A., Bruni-Cardoso A., Augusto T. M. (2018). Macrophage roles in the clearance of apoptotic cells and control of inflammation in the prostate gland after castration. *The Prostate*.

[20] Korfage I. J., de Koning H. J., Roobol M., Schroder F. H., Essink-Bot M. L. (2006). Prostate cancer diagnosis: the impact on patients’ mental health. *European Journal of Cancer*.

